This article has been retracted.

# Analysis of Hazard Factors Affecting the Quality of Life for Lung Cancer Patients after Chemotherapy

**DOI:** 10.1155/2022/6910126

**Published:** 2022-04-20

**Authors:** Lianying Wen, Xiaohong Liao, Yanjin Cao, Yanxiu Liu, Wei Wu, Yan Chen, Huiyu Liu

**Affiliations:** ^1^Department of Respiratory and Critical Care Medicine, Ganzhou People's Hospital, 16 Meiguan Avenue, Ganzhou 341000, Jiangxi, China; ^2^Department of Otolaryngology, Ganzhou People's Hospital, Ganzhou 341000, Jiangxi, China

## Abstract

**Objective:**

To explore the hazard factors affecting the quality of life for patients with lung cancer after chemotherapy, so as to provide evidence-based clinical proof to improve their quality of life.

**Methods:**

The clinic data of lung cancer patients treated with chemotherapy from November 2020 to November 2021 in our hospital were selected for retrospective analysis. A questionnaire survey was administered to 74 patients who met the inclusion criteria. The general condition questionnaire made by the department was used to analyzed the patients' demographic characteristics and disease status. The *quality of life questionnaire for Chinese cancer patients receiving chemobiotherapy* (QLQ-CCC) was used to evaluate the patients' quality of life.

**Results:**

The research objects selected for this study scored an average of (94.53 ± 22.65) points in the quality of life. It was found by logistic regression analysis that age, education level, marital status, pathological types, monthly family income, and metastasis were the independent influencing factors that lowered the quality of life of lung cancer patients after chemotherapy (*P* < 0.001).

**Conclusion:**

Chemotherapy can lead to a decline in the quality of life of lung cancer patients, and there are many factors at play. Therefore, medical and nursing staff should focus on the overall condition of patients when carrying out clinical treatment.

## 1. Introduction

Lung cancer is currently the leading cause of death from malignancies worldwide [1], with a 5-year survival rate of less than 20% and approximately 730,000 new cases per year. Lung cancer is mainly divided into non-small-cell lung cancer and small cell lung cancer [2, 3]. The cause of lung cancer remains unclear and may be related to smoking, air pollution, ionizing radiation, and genetics. At present, the preferred treatment protocol for lung cancer is an integrated therapy based on surgical resection. But for advanced patients who have lost the chance to receive surgery, the 5-year survival rate is less than 25%. The treatment modalities for advanced lung cancer mainly include chemotherapy, targeted therapy, immunotherapy, radiotherapy, and traditional Chinese medicine treatment. Chemotherapy is the primary tool for curing lung cancer, which means using chemical drugs to kill cancer cells so as to control tumor growth [4, 5]. However, since chemotherapy is systemic and not targeted, it causes harm to normal cells while killing cancer cells, and brings about serious side effects such as nausea, vomiting, and depression while prolonging the survival time and relieving physical pain of patients [6]. As the economy develops, the expectation of cancer patients for treatment is no longer just to prolong their survival time, but to obtain a higher quality of life. With the new contemporary understanding of health, traditional evaluation indexes such as survival time and clinical efficacy cannot meet the demands for comprehensive assessment of efficacy [7], so the quality of life has gradually been applied to medicine. Due to the late start of research on quality of life in China, there are few research into the quality of life after chemotherapy in cancer patients [8]. The quality of life questionnaire is an important channel to know and study the quality of life for patients [9]. Patients' quality of life after chemotherapy is not only affected by the body but also changes with the mentality, and there are plenty of complicated factors that can make a difference [10]. Therefore, we conducted a retrospective analysis of the hazard factors affecting the quality of life for patients after chemotherapy by launching a questionnaire survey of the quality of life for the research objects in this study. It is expected to provide more evidence-based proof for the selection and prognosis of cancer treatments and bring more benefits to patients with malignant tumor diseases.

## 2. Materials and Methods

### 2.1. General Data

The research objects selected for this study were the lung cancer patients who received chemotherapy treatment from November 2020 to November 2021 in our hospital. The study was in line with the Declaration of Helsinki (2013) [11]. The inclusion criteria were as follows: (1) the patients met the diagnostic criteria of the *Chinese Medical Association guidelines for clinical diagnosis and treatment of lung cancer* [12] *(edition 2018)* and were confirmed by MRI, CT, and histopathological examination, with symptom manifestations of cough, hemoptysis, pleural effusion, and dysphagia; (2) the patients were eligible for chemotherapy (with normal indexes of liver function, blood routine, and renal function and without other serious complications), and their performance status scores (KPS) were no less than 60; and (3) the patients had no other comorbidities that obviously threatened their quality of life except for the primary disease, lung cancer.

The exclusion criteria were as follows: (1) patients with major diseases such as liver, kidney, brain, and heart dysfunctions; (2) patients with communication or comprehension disturbance that make it difficult to cooperate with the scale assessment; (3) patients who switched to other treatment regimens during chemotherapy; and (4) patients with psychiatric symptoms and previous oral medications of sedative and antidepressant drugs.

### 2.2. Methods

#### 2.2.1. Investigation Tools

In this study, the questionnaires included general condition and quality of life questionnaires.

#### 2.2.2. General Condition Questionnaire

The questionnaire was designed by the department, mostly including gender, age, pathological types, family income, and residence of the patients.

#### 2.2.3. Quality of Life Questionnaire

The *quality of life questionnaire for Chinese cancer patients with chemobiotherapy* (QLQ-CCC) [13] was adopted to assess the quality of life for lung cancer patients. The patients completed the questionnaire, then handed it to the researcher, and the score was calculated uniformly and input into the computer. The scale was a closed-ended questionnaire consisting of 35 entries in 4 areas which were physical (16 questions), mental and psychological (5 questions), social (5 questions), and other aspects (9 questions). The responses were a combination of numerical ratings and written descriptions. Each question had 5 alternative answers rated on a scale of 1–5, with a total score of 35–175. The higher the score, the better the quality of life. The internal consistency coefficient of the scale was 0.862, and all the correlation coefficients were *P* < 0.001.

### 2.3. Distribution of the Questionnaires

The questionnaires were issued by the researcher who specified how to fill in the scale to the respondents with uniform instructions. The respondents were required to complete the questionnaires independently within 45 min, and the questionnaires were retrieved as soon as they were finished.

### 2.4. Statistical Methods

Professional statistical software SPSS 26.0 was used to process the data of this study. The patients' quality of life was evaluated by total scores, mean scores, and standard deviations. Logistic regression was used to analyze the effects of demographic factors and disease factors on the quality of life for lung cancer patients after chemotherapy, and *P* < 0.05 indicated that the differences were statistically significant.

## 3. Results

### 3.1. QLO-CCC Results of Patients

The results are shown in Table 1.

### 3.2. Univariate Analysis of Factors Affecting Quality of Life for Lung Cancer Patients after Chemotherapy

The results are detailed in Table 2.

### 3.3. Logistic Regression Analysis of Factors Affecting the Quality of Life

Taking the QLQ-CCC scores as the dependent variables, the univariates with statistical significance were included in the multivariate logistic regression analysis which concluded that age, education levels, marital status, pathological types, monthly family income, and metastasis were independent influencing factors lowering the lung cancer patients' quality of life after chemotherapy, as shown in Table 3.

## 4. Discussion

Lung cancer is a malignant tumor with high morbidity and mortality in China, which not only threatens the physical and mental health of patients, but also is a menace to their lives [14]. In recent years, with the advances in medical technology, the morbidity and mortality of lung cancer remain high, which has become a major public health issue in China [15]. As a common treatment for lung cancer, chemotherapy can keep the condition under control and mitigate clinical symptoms effectively. However, most of these drugs have high cytotoxicity, which not only kill cancer cells but also damage normal cells and tissues of the body, causing adverse effects on the daily life and psychology of patients [16]. In the past, the effectiveness assessment of treating lung cancer only put emphasis on the change of tumor size, survival time, and metastasis, instead of patients' quality of life.

Quality of life refers to the overall feeling of people thinking about their individual health and state of life, which is mostly evaluated from the physical, psychological, and social aspects of patients in medicine [17]. There are lots of factors affecting the quality of life of lung cancer patients after chemotherapy such as pathological types and age. Besides, studies [18] have found that underlying diseases and pathological stages might also have an impact. In this study, lung cancer patients admitted to our hospital were selected as research objects. It was found by multivariate logistic regression analysis that age, education levels, marital status, pathological types, monthly family income, and metastasis were the independent influencing factors exacerbating the decline of their quality of life.

It has been found that after chemotherapy, the older the patients are, the poorer their physical functions are, which is due to the fact that the physiological functions of vital organs such as the liver and kidney, as well as the generation and reserve capacity of bone marrow decline gradually along with age. Therefore, the tolerance to chemotherapy will diminish, resulting in a poor quality of life after chemotherapy [19]. As a result, the risks and benefits of receiving chemotherapy should be evaluated with caution for elderly patients, and the observation and nursing care of patients' conditions should be intensified during treatment. The results of this study showed that the QLQ-CCC scores were higher in patients with a college degree or above than in patients with a high school degree or below. Probably because patients with higher degrees tend to actively understand and seek information about diseases and therapy, use their social support effectively, and coordinate with treatment. For chemotherapy patients with lower education levels, nurses should take the initiative to communicate with them and offer health education in plain language and efficient social support in order to improve their treatment compliance [20]. Marital status is also an important factor that may decline lung cancer patients' quality of life after chemotherapy. This study found that the QLQ-CCC scores were significantly higher in married patients than in unmarried and divorced patients, because single patients lack spiritual support from their families to withstand diseases. Harmonious family ties can make patients feel loved, and mental comfort alleviates the cancer pain to some extent, resulting in a better quality of life [21]. In terms of pathological types, patients with non-small-cell lung cancer had a far better quality of life than those with small cell lung cancer. That is because, with a high degree of malignancy, rapid cell growth and an early metastasis, small cell lung cancer often metastasizes to the liver, brain, bone, and other organs. Patients with metastasis have a late clinical stage and therefore a poor prognosis [22]. Economic status is one of the main factors that works as well, and patients in worse economic conditions tend to have a lower quality of life. Because patients who have undergone multiple chemotherapy may develop many toxic and adverse reactions and their physical functions are at poor levels, for which reason they need more drugs to lessen the side effects, followed by a spike in medical expenses. The expensive chemotherapy drugs increase the family burden of patients and deteriorate their financial situations. Therefore, medical workers are supposed to focus on the family income of patients. Especially for those suffering economic hardship, effective measures and preferential policies need to be conducted to ease their burdens [23, 24]. Whether the cancer has metastasized is also an essential factor affecting the patients' quality of life. Some studies have found that patients who have a higher number of organs with metastatic tumors have a poorer quality of life and more obvious symptoms such as pain, cough, and panting, which are considered to be related to the damage of their organs with metastatic tumors. Therefore, medical and nursing staff should strengthen the clinical monitoring of patients with metastasis [25].

The limitations of this study are as follows: due to the single sample source, small sample size, and deficient or inadequate considerations about the factors affecting patients' quality of life after chemotherapy, the study results lacked universality and systematicness. In addition, the influences from chemotherapy regimens on patients' quality of life were not considered. The investigations into nutritional status, chemotherapy regimens, and beliefs should be added in future research studies to observe their impacts on patients' quality of life. Thus, researchers can fully understand the factors affecting lung cancer patients' quality of life after chemotherapy and explore methods for improving their quality of life.

## Figures and Tables

**Table 1:** QLQ-CCC results of lung cancer patients.

Items	Score range	Minima	Maxima	Mean scores
Physical aspect	16–80	23	56	39.05 ± 9.91
Mental and psychological aspects	5–25	8	18	12.91 ± 3.18
Social aspect	5–25	9	16	12.42 ± 2.46
Others	9–45	14	32	22.47 ± 5.42
Total scores	35–175	56	134	94.53 ± 22.65

**Table 2:** Univariate analysis of factors affecting quality of life for lung cancer patients after chemotherapy.

Items	n	QLQ-CCC scores	t	*P*
*Gender*				
Male	46	123.74 ± 11.89	7.929	<0.001
Female	28	102.18 ± 10.37		

*Age*				
25−45	8	131.50 ± 1.60	13.677	<0.001
46−60	26	92.81 ± 9.36		
>60	40	66.90 ± 9.65		

*Education levels*				
College or above	9	131.00 ± 2.00	9.579	<0.001
High school	20	101.65 ± 18.37		
Middle school or below	45	70.44 ± 11.48		

*Career*				
Staff members	14	91.64 ± 21.71	0.140	0.890
Farmers	19	90.11 ± 21.93		
Workers	25	90.60 ± 21.13		
Individual business owners	16	88.88 ± 22.51		

*Lesion locations of tumor*				
Central types	35	97.77 ± 22.27	1.176	0.244
Peripheral types	39	91.72 ± 21.94		

*Marital status*				
Married	5	84.80 ± 17.20	9.419	<0.001
Unmarried	62	120.58 ± 7.66		
Divorced	7	90.57 ± 7.16		
Pathological types				
Small cell lung cancer	23	91.04 ± 16.27	12.347	<0.001
Non-small-cell lung cancer	51	123.27 ± 6.25		

*Payment methods*				
Self-paying	14	100.64 ± 22.40	0.473	0.655
Medical insurance	31	95.39 ± 23.30		
Cooperative medical service	29	95.41 ± 22.90		

*Monthly family income*				
≥3000	39	127.67 ± 3.74	18.399	<0.001
<3000	35	91.37 ± 11.68		

*Metastasis*				
Yes	23	90.83 ± 15.03	14.982	<0.001
No	51	126.31 ± 5.35		

*Residence*				
Rural area	40	90.33 ± 22.30	0.192	0.848
Urban area	34	91.38 ± 24.64		

**Table 3:** Logistic regression analysis of factors affecting the quality of life.

Factors	Β	Se	Wald	*P*	OR	OR 95% CI
Gender	0.731	0.471	8.273	0.241	1.253	1.012–1.516
Age	0.261	0.062	6.381	<0.001	4.328	3.819–5.213
Education levels	0.327	0.723	2.371	0.021	3.212	2.972–3.988
Marital status	1.253	1.923	3.267	<0.001	2.361	1.832–3.021
Pathological types	1.317	1.025	4.182	<0.001	3.283	2.734–4.327
Monthly family income	0.531	0.371	12.381	0.025	8.821	7.361–9.298
Metastasis	2.072	0.512	9.283	0.009	0.253	0.134–0.482

## Data Availability

The data to support the findings of this study are available on reasonable request from the corresponding author.
